# Brain Network for Exploring the Change of Brain Neurotransmitter 5-Hydroxytryptamine of Autism Children by Resting-State EEG

**DOI:** 10.1155/2022/5451277

**Published:** 2022-04-23

**Authors:** Jun Shao, Fan Zhang, Chuanzhi Chen, Ye Wang, Qiang Wang, Jie Zhou

**Affiliations:** ^1^Department of Physical Diagnostics, Hongqi Hospital Affiliated to Mudanjiang Medical University, Mudanjiang, 157000 Heilongjiang, China; ^2^Department of Heilongjiang Key Laboratory of Antifibrosis Biotherapy, Mudanjiang Medical University, Mudanjiang, 157000 Heilongjiang, China; ^3^Department of Nuclear Medicine, Hongqi Hospital Affiliated to Mudanjiang Medical University, Mudanjiang, 157000 Heilongjiang, China; ^4^Department of Cardiology, Mudanjiang Medical University, Second Affiliated Hospital, Mudanjiang, 157000 Heilongjiang, China; ^5^Department of Fever Clinics, Hongqi Hospital Affiliated to Mudanjiang Medical University, Mudanjiang, 157000 Heilongjiang, China

## Abstract

The study was aimed at understanding the brain network and the change rule of brain neurotransmitter 5-hydroxytryptamine (5-HT) in autism children through resting-state electroencephalogram (EEG). 20 autistic children in hospital were selected and defined as the observation group. Meanwhile, 20 healthy children were defined as the control group. EEG signals were collected for the two groups. Fuzzy C-means (FCM) algorithm was used to extract features of EEG signals, and DTF was applied for the causal association between multichannel EEG signals. The two groups were compared for the average function value and regional efficiency of the brain neurotransmitter 5-HT. The results showed that the classification accuracy of frontal F7 channel, left frontal FP1 channel, and temporal T6 channel was 95.2%, 95.3%, and 91.2%, respectively. The average of high beta frequency band, low beta frequency band, theta frequency band, and alpha frequency band in the control group was significantly higher than that in the observation group under the optimal threshold (*P* < 0.05). Compared with normal subjects (34.27), the average function of 5-HT in the brain was 20.13 in patients with low function and 45.74 in patients with hyperfunction. In conclusion, FCM algorithm can feature extraction of EEG signals, especially in the frontal F7 channel, the left frontal FP1 channel, and the TEMPORAL T6 channel, which has high classification accuracy and can well express the EEG signals of autistic children. The level of 5-HT in autistic children is lower than that in healthy people, and it is closely related to loneliness and depression.

## 1. Introduction

Autism is a neurodevelopmental disorder associated with impairment of executive function, language, emotion, and social function [1–3]. Autistic children show very different levels of intelligence, with a few patients in the normal range and most of them with different degrees of intellectual impairment. Studies have shown that about 50% of autistic children have moderate or above intellectual deficiency (IQ less than 50), 25% have mild intellectual deficiency (IQ between 50 and 69), and 25% have normal intelligence (IQ greater than 70). Those with normal intelligence are called high-functioning autism [4–7].

The causes of autism are still unknown, but the main influencing factors include perinatal factors, genetics, immune system abnormalities, neuroendocrine, and neurotransmitters. The role of genetic factors on autism tends to be clear, but the specific genetic mode has not been specifically identified [8, 9]. With regard to the immune system, scholars have found that the decrease of T lymphocytes, helper T cells, and B cells, the decrease of natural killer cell activity, and the lack of inhibition-induction T cells are all related to autism. The dysfunction of neurotransmitters will affect neuroendocrine system. The monoamine system of patients with autism, such as 5-hydroxytryptamine (5-HT) and catecholamine, is immature, and the abnormal pineal gland-hypothalamus-pituitary-adrenal axis will lead to the increase of 5-HT and endorphin and the decrease of ACTH secretion [10, 11]. Selective 5-HT reuptake inhibitor is effective for the behavioral and emotional problems of patients with autism. However, the drugs are still insufficient in improving patients' behaviors. Early education, training, and behavioral intervention for autism children can effectively improve children's development and their quality of life [12, 13].

Doppler examination can judge cerebrovascular velocity, blood vessel elasticity, and blood vessel size. Judging the blood flow velocity can identify whether there is vasospasm, whether there is plaque in the blood vessel, and whether there is vascular stenosis [14, 15]. Electroencephalogram (EEG) can present the neurobiological signal changes related to postsynaptic potentials of cerebral cortex, mainly brain activity and complex nerves. It is a powerful tool to research mental illnesses. There have been studies exploring the biological phenotype of autism patients from the brain structure and function level. Evoked potentials reflect the electrophysiological changes of the greater brain nerve in the cognitive process [16]. EEG signals are nonlinear coupled by a large number of neurons and are highly nonlinear multiunit connected aggregates. In the absence of external stimuli or cognitive tasks, the cerebral cortex is still busy with complex neuronal discharges. This spontaneous activity state is called the resting state, and the resting-state EEG signals can reflect the information integration and new processing process. Complex brain network can effectively integrate information globally. Autism children are too young, and it is difficult to collect EEG in task state. Thus, EEG research in resting state has stronger advantages. The establishment of brain functional network mainly relies on functional magnetic resonance imaging, EEG, magnetoencephalography, and other imaging technologies [17]. Fuzzy C-means clustering (FCM) algorithm is widely used in pattern recognition, image processing, and fuzzy modeling, because it can optimize the brain image segmentation method [18].

Nowadays, FCM has been widely used in medical diagnosis, image analysis, agricultural environmental engineering, and target recognition. Especially, image processing can reduce image noise, which has important guiding significance for the analysis and research of medical images. Based on resting-state EEG, this study analyzed the brain network of patients with autism and discussed the change rule of 5-HT, to understand the differences of track the characteristics of brain function changes, expected to provide a theoretical basis for preventing the occurrence of autism. This study hoped that the FCM algorithm has certain application value in EEG imaging and provides a reference for clinical EEG analysis.

## 2. Materials and Methods

### 2.1. Clinical Data

In this study, 20 autistic children from June 2019 to December 2020 were selected, including 11 boys and 9 girls. The mean age was 1.6 ± 1.9 years. All patients were diagnosed according to the *Diagnostic and Statistical Manual of Mental Disorders* (4th edition). Parents who filled in the Autism Behavior Scale (ABC) scored more than 62. Further, 20 healthy children during the same period were selected as the control group according to the principle of race, age, sex, and education level similar to the observation group. Among the 20 healthy volunteers, 8 were boys and 12 were girls, with an age range of 1.5-1.8 years. All data came from the EEG at the Children's Hospital. All patients who fully met the inclusion criteria accepted the trial regulations and signed the informed consent for the experiment. The study had been approved by the ethics committee of hospital.

Inclusion criteria are as follows: (1) the first onset of autism; (2) stable basic vital signs, verbal expression, and clear consciousness; (3) no history of head trauma; (4) no neurological diseases or other mental disorders; (5) no visual impairment and EEG contraindications; and (6) right handedness. Exclusion criteria are as follows: (1) with a history of drug dependence, abuse, and alcoholism; (2) previous manic episodes; (3) mental retardation; (5) unable to accept EEG examination due to their own reasons; and (6) incomplete clinical data.

### 2.2. EEG Acquisition

All scans are performed in hospital. 128-guide EEG acquisition system is used to collect resting-status EEG in 5 minutes. The sampling rate is set to 1000 Hz, and the impedance of the set is less than 50 k*Ω*. During sampling, the child quietly sat in front of the screen at 80 cm, kept relaxed, and breathed evenly. With the head still as much as possible, the child was guided to watch bubbles and small fish moving slowly on the screen. EEG collection process is based on 10-20 system electrode placement, as shown in Figure 1.

Figure 1 (a) The lateral face from FPzJ to Oz through T3 and T4, with the total length of 100%, respectively. The left frontal pole (FP1) and right frontal pole (FP2) are 10% from left and right of FPz; the left occipital point (O1) and right occipital point (O2) are 10% from left and right of Oz. The left front point (F7, F8) is the midpoint of FP1 and T3 and the midpoint of FP2 and T4. The right posterior point (T5, T6) is the midpoint of O1 and T3 and the midpoint of O2 and T4. (b) The left and right frontal points (F3, F4) are the midpoints of FP1 and C3, FP2 and C4, or between Fz and F7 and F8, while the left and right vertices (P3, P4) are between C3 and O1, C4 and O2, or between Pz and T5 and T6.

The EEG at the resting state of the children is collected under the condition of open eyes, and the scan lasts no less than 20 minutes. The doctor should keep the environment quiet to avoid environmental interference. The behavior state of the children is recorded synchronously in the form of video. Unipolar, transverse, longitudinal, and cyclic analyses are performed in each case. Each time, the result is judged by two people. Before data collection, professional personnel will assess the scan safety of the subjects. After confirming that there are no contraindications, detailed inspection procedures and precautions will be introduced.

Unified guidance for image acquisition: the subject tries to keep his head still during the scanning process. The doctor carefully observes the scanned image data; and the image data that does not meet the requirements such as the data with larger head movement is removed, to ensure data quality in every step of data processing and to eliminate noises and other confounding factors.

### 2.3. TCD Doppler Detection

Color Doppler diagnostic instrument is used to measure the mean velocity and resistance index of a large number of arteries through temporal window. EEG examination is performed according to the *Clinical Odeon Tutu Criteria*.  Table 1 shows the reference standard values of brain neurotransmitters.

### 2.4. Structure of the Brain Network

There are great differences in clinical symptoms. Some markers do not provide a reasonable explanation for the great symptom heterogeneity of patients. The brain network graph theory based on the structural and functional neuroimaging provides a new idea to understand and explain this phenomenon. The brain network realizes the interaction between brain regions through connection. Each network consists of nodes (brain regions) connected by edges (connections between nodes). Brain networks can be constructed using structural and functional neuroimaging data. In structured imaging, the connection between nodes can be realized by diffusion tensions, thus representing anatomical link between individual nodes. In functional imaging, the connection of nodes is based on their correlation with MRI blood oxygen level-dependent time series. There may or may not be structural support between functional connection areas. The brain regions with related activities are likely to form a network (Figure 2).

### 2.5. FCM Algorithm

Cluster analysis is a mathematical method to classify similar data points in a sample set according to a specific criterion. The purpose is to classify a group of labeled vectors in a specific space into several subsets according to some similarity criteria. The steps of cluster classification include (1) feature extraction and selection of cluster objects, (2) definition of similarity measure function, (3) clustering, and (4) evaluation of results.

If samples in *A* = {*X*1, *X*2, ..Xi, ⋯Xn} are classified as *C*, and *C* is a positive integer > 1, then any local point *Xi* ∈ *X*(1 ≤ *i* ≤ *n*).

The degree of *X*_*j*_ ∈ *X*(1 ≤ *j* ≤ *n*) is expressed as *K*_*ji*_ (1 ≤ *K*_*ji*_ ≤ 1), the fuzzy clustering of sample space *X* is described by fuzzy matrix *K* = *K*_*ji*_, and the element in the *i*th of *j*th column of matrix *K* is expressed as *K*_*ji*_ to represent the membership degree of the *i*th sample point belonging to the *j* class. The properties of *K* are as follows.

(1) $$\begin{array}{c} K_{ji}=\in \left[0,1\right], \end{array}$$

(2) $$\begin{array}{c} \overset{\text{c}}{\underset{j=1}{\sum }}K\text{ij}=1, \end{array}$$

(3) $$\begin{array}{c} 0<\overset{\text{c}}{\underset{j=1}{\sum }}K\text{ij}=<\text{n}. \end{array}$$

FCM algorithm is used to calculate the membership degree of each point relative to the clustering center, and the objective function is expressed as follows.

(4) $$\begin{array}{c} J\text{m}\left(W,H\right)=\overset{n}{\underset{i=1}{\sum }}\overset{c}{\underset{j=1}{\sum }}{w^{m}}_{ij}{d^{2}}_{ij}\left(x_{i},k_{j}\right),\;\text{h}=\left(h_{1},h_{2},h_{3}\cdots h_{c}\right), \end{array}$$

where *h*_*j*_ represents the clustering center of the *j*th class and *m* (*m* > 1) is a fuzzy function.

(5) $$\begin{array}{c} {{\text{d}}^{2}}_{ij}\left(x_{i},h_{j}\right)=\left\|\text{x}i-h\text{j}\right\|. \end{array}$$

Equation (5) is the Euclidean distance from sample point *X*_*i*_ to cluster center *H*_*j*_.

FCM realizes fuzzy classification of sample set by iterative optimization of objective function.

1. Random initialization of *M*^(0)^. *U*^(0)^ is initialized and *M*^(0)^ is calculated. The number of iterations is *n* = 1, the number of clustering centers is *C*, and the fuzzy index is *m* (*m* > 1)
2. Calculation of M(n). If ^∀^ *i* and *r* and *d*^*ir*^(*n*) > 0, then the equation below is obtained.

(6) $$\begin{array}{c} M\text{ij}=\frac{1}{\sum_{r=1}^{c}\left[{\left(d_{ij}\left(n\right)/d_{ir}\left(n\right)\right)}^{2/m-1}\right]} \end{array}$$

(3) Calculation of *H*^(*n* + 1)^, ^∀^*j*.

(7) $$\begin{array}{c} H_{\text{j}}\left(n+1\right)=\frac{\sum_{i=1}^{n}{M^{m}}_{ij}x_{i}}{\sum_{i=1}^{n}{M^{m}}_{ij}} \end{array}$$

(4) If the ‖*M*(*n*) − *M*(*n* + 1)‖ < *δ*, the iteration is stopped. Otherwise, *n* = *n* + 1, and return to the step (2). *δ* is a pregiven small positive number. FCM largely depends on the selection of the initial clustering center. When the initial clustering center deviates seriously from the global optimal clustering center, the algorithm will fall into the local minimum

### 2.6. Frequency Domain Causal Analysis

EEG reflects the temporal correlation between functional signals of brain conductance. Granger causality test does not require prior knowledge and is superior to other methods. In the analysis of time series, Granger causality test establishes binary linear equation, and directional transfer function (DTF) is used for multiple regression model. In this study, DTF is applied in the causal relationship between multichannel EEG signals, and the time series of 19-channel EEG signals are as follows.

(8) $$\begin{array}{c} X\left(\text{t}\right)={\left[x_{1}\left(t\right),x_{2}\left(t\right)\cdots x_{19}\left(t\right)\right]}^{T}. \end{array}$$

The multiple regression model is expressed as follows.

(9) $$\begin{array}{c} \overset{\text{n}}{\underset{k=0}{\sum }}B\left(K\right)X\left(t-k\right)=E\left(t\right). \end{array}$$

*N* represents the order of the model, and *B*(*K*) is the model coefficient matrix of 19 × 19. *A*(0) = *H*, *H* is the identity matrix, and *E*(*t*) is the multivariate standard white noise vector.

The conversion frequency domain equation is as follows.

(10) $$\begin{array}{c} B\left(f\right)X\left(f\right)=E\left(f\right), \end{array}$$

where

(11) $$\begin{array}{c} B\left(f\right)=\overset{n}{\underset{k=0}{\sum }}B\left(K\right)e^{-j2\pi \text{fk}}. \end{array}$$

Then,

(12) $$\begin{array}{c} X\left(f\right)={\text{B}}^{‐1}\left(f\right)E\left(f\right)=G\left(f\right)E\left(f\right). \end{array}$$

*G*(*f*) represents the transfer matrix, so the causal connection *β*_sq_(*f*) of channel *s* to *q* is as follows.

(13) $$\begin{array}{c} {\beta^{2}}_{\text{sq}}\left(f\right)=\frac{{\left|G_{\text{sq}}\left(f\right)\right|}^{2}}{\sum_{\text{m}=1}^{K}{\left|G_{\text{sq}}\left(f\right)\right|}^{2}}. \end{array}$$

There is causality between multiple channels, and DTF can calculate the Granger causality between multiple channels. In this study, the 95% confidence interval *β*_sq_(*f*) is 0. *β*_sq_ in DTF matrix is evaluated, and nonparametric test is carried out between the initial DTF matrix and the empirical distribution of the recombined data.

### 2.7. Statistical Methods

SPSS22.0 is used for experimental data processing, and analysis methods are selected according to different conditions. Single factor analysis and *χ*^2^ test are employed to represent the mean ± standard deviation of data. EEG data of the two groups are cut into 30 segments during the establishment of brain network. *P* < 0.05 is considered statistically different.

## 3. Results

### 3.1. EEG Images

In Figure 3, (a) is the beta wave, (b) is the alpha wave, (c) is the theta wave, and (d) is the delta wave. Figures 4 and 5 are the fast and slow waves within 1 second.

### 3.2. Classification Results of EEG

As shown in Table 2, the classification accuracy of frontal F7 channel, left frontal FP1 channel, and temporal T6 channel was 95.2%, 95.3%, and 91.2%, respectively, when FCM algorithm was used for EEG classification and recognition. Different brain regions have different functions. EEG abnormalities in the frontal lobe indicate poor cognitive ability of children, while abnormalities in the temporal region indicate language and social disorders. These characteristics are consistent with the characteristics of autism children.

### 3.3. Whole-Brain Local Efficiency

Figure 6 shows the average of children's network in high beta band, low beta band, theta band, and alpha band under the optimal threshold, and the control group was significantly higher than the observation group in each band (*P* < 0.05).

### 3.4. 5-HT Function Distribution

Figure 7 shows the function values of 5-HT in the observation group and the control group. Compared with normal subjects (34.27), the average function of 5-HT in the brain was 20.13 in patients with low function and 45.74 in patients with hyperfunction. The mean function of 5-HT in high-functioning patients was significantly higher than the distribution of 5-HT in normal subjects and low-functioning patients (*P* < 0.05).

## 4. Discussion

The number of autism patients is increasing, and it has a serious impact on the quality of life of patients. EEG signals record the electrophysiology of the cerebral cortex and identify the electrical characteristics of the brain in children. Local consistency indicators in resting-state EEG have many advantages of high stability, good patient compliance, high repeatability, and avoidance of potential performance confounding factors related to cognitive activation in task-based MRI [19, 20]. EEG is a well-established and noninvasive tool for neurophysiological characterization and monitoring of electrical activity in the brain. It can identify abnormalities associated with the frequency range, connectivity, and lateralization of brain function. Different genetic and environmental etiologies result in autism spectrum disorders, which manifests at the macro level as abnormal neural connections. Previous studies have described the dynamics of neural oscillations within the atypical mode *α* range (6-12 Hz) of the reduction of short and medium distance connections and the increase of long-distance connections and found that it was sensitive to the healthy development of functional and structural connections. Therefore, EEG with high temporal accuracy is an ideal tool for studying neural connectivity in developing populations. Dickinson et al. (2018) [21] tested spontaneous *α* phase consistency in heterogeneous samples of 59 autistic children and 39 age-matched typically developing children. They used the data-driven approach to perform unbiased examination of all possible atypical connectivity patterns in all cortical regions. The temporal low connectivity between the hemispheres of the brain represents fundamental functional differences in children with autism and may reflect white matter disorders or increased temporal signal variability in children with autism. Reis Paula et al. (2017) [22] showed that the frontal lobe, central lobe, parietal lobe, and occipital lobe regions were highly activated at higher frequencies (above 30 Hz) in the atrioventricular deficiency group. This may be related to the developmental characteristics of children with autism. Reduced connectivity between brain regions is thought to be responsible for autism symptoms. Pillai et al. (2018) [23] showed enhanced connectivity in children with autism. It may be that behavioral changes in brain connections are more important than absolute differences in autism connections. The results of this study showed that the classification accuracy of frontal F7 channel, left frontal FP1 channel, and temporal T6 channel was above 90% in EEG classification. Different brain regions have different functions. EEG abnormalities in the frontal lobe indicate poor cognitive ability of children, while abnormalities in the temporal region indicate language and social disorders. These characteristics are consistent with the characteristics of autism children.

As a brain neurotransmitter in the central nervous system, 5-HT plays a very important role in regulating human emotions. And 5-HT receptors play an important role in the pathogenesis of depression and the mechanism of action of antidepressants. It is known that there are at least seven 5-HT receptors in humans, and most of them have been cloned [24]. Dysfunction of the 5-HT system can lead to a variety of psychiatric disorders, including depression, anxiety, obsessive-compulsive disorder, autism, and eating disorders. The availability of human i5HT neurons will be very useful for research and drug discovery in many serotonin-related psychiatric disorders [25]. The results of this study showed that compared with normal subjects (34.27), the average function of 5-HT was 20.13 in patients and 45.74 in patients with hyperfunction. FCM algorithm was used to classify the EEG features of children, and the accuracy of each channel showed that the rhythm waves with different frequencies could classify the brain features well.

## 5. Conclusion

The study was aimed at understanding the brain network and the change rule of 5-HT in autism children through resting-state EEG. 20 autistic children were selected and defined as the observation group. Meanwhile, 20 healthy children were defined as the control group. EEG signals were collected for the two groups. FCM algorithm was used to extract features of EEG signals, and DTF was applied for the causal association between multichannel EEG signals. The two groups were compared for the average function value and regional efficiency of the brain neurotransmitter 5-HT. FCM algorithm can feature extraction of EEG signals, especially in the frontal F7 channel, the left frontal FP1 channel, and the temporal T6 channel, which has high classification accuracy, and can well express the EEG signals of autistic children. The level of 5-HT in autistic children is lower than that in healthy people, and it is closely related to loneliness and depression. However, some limitations in the study should be noted. The sample size is small, which will reduce the power of the study. In the follow-up, an expanded sample size is necessary to strengthen the findings of the study. All in all, the FCM algorithm used in this study provides EEG signals, which is worthy of clinical promotion and has a certain reference value.

## Figures and Tables

**Figure 1:** 10-20 system electrode placement.

**Figure 2:** Schematic diagram of brain network structure.

**Figure 3:** Different frequency band.

**Figure 4:** Fast wave.

**Figure 5:** Slow wave.

**Figure 6:** The average of brain network under optimal threshold. # represents significant difference, *P* < 0.01; ∗ represents significant difference, *P* < 0.05.

**Figure 7:** Function distribution of 5-HT. ∗ represents significant difference, *P* < 0.05.

**Table 1:** Brain neurotransmitter.

Neurotransmitter	Homogeneity	Standard deviation (S)	Hyperfunction	Low function
5-HT	16.256	3.784	>37.473	<30.225

**Table 2:** Classification results of EEG.

Aisle	Accuracy	Aisle	Accuracy
C3	87.5%	O1	89.1%
C4	86.2%	02	82.5%
F3	89.3%	P3	79.8%
F4	89.3%	P4	86.3%
F7	95.2%	T3	82.8%
F8	88.4%	T4	89.5%
FP1	95.3%	T5	89.6%
FP2	86.5%	T6	91.2%

## Data Availability

The data used to support the findings of this study are available from the corresponding author upon request.
